# Examination of validity, reliability, and interpretability of a self-reported questionnaire on Occupational Balance in Informal Caregivers (OBI-Care) – A Rasch analysis

**DOI:** 10.1371/journal.pone.0261815

**Published:** 2021-12-23

**Authors:** Anna Röschel, Christina Wagner, Mona Dür

**Affiliations:** 1 Department of Health Sciences, IMC University of Applied Sciences Krems, Krems, Austria; 2 Duervation, Krems, Austria; Sunway University, MALAYSIA

## Abstract

**Objectives:**

Informal caregivers often experience a restriction in occupational balance. The self-reported questionnaire on Occupational Balance in Informal Caregivers (OBI-Care) is a measurement instrument to assess occupational balance in informal caregivers. Measurement properties of the German version of the OBI-Care had previously been assessed in parents of preterm infants exclusively. Thus, the aim of this study was to examine the measurement properties of the questionnaire in a mixed population of informal caregivers.

**Methods:**

A psychometric study was conducted, applying a multicenter cross-sectional design. Measurement properties (construct validity, internal consistency, and interpretability) of each subscale of the German version of the OBI-Care were examined. Construct validity was explored by assessing dimensionality, item fit and overall fit to the Rasch model, and threshold ordering. Internal consistency was examined with inter-item correlations, item-total correlations, Cronbach’s alpha, and person separation index. Interpretability was assessed by inspecting floor and ceiling effects.

**Results:**

A total of 196 informal caregivers, 171 (87.2%) female and 25 (12.8%) male participated in this study. Mean age of participants was 52.27 (±12.6) years. Subscale 1 was multidimensional, subscale 2 and subscale 3 were unidimensional. All items demonstrated item fit and overall fit to the Rasch model and displayed ordered thresholds. Cronbach’s Alpha and person separation index values were excellent for each subscale. There was no evidence of ceiling or floor effects.

**Conclusions:**

We identified satisfying construct validity, internal consistency, and interpretability. Thus, the findings of this study support the application of the German version of the OBI-Care to assess occupational balance in informal caregivers.

## Introduction

Persons with an impairment or a disease, such as preterm infants or persons with dementia, rely on the support and care of informal caregivers. Informal caregivers are defined as close family members, relatives or friends that provide unpaid care [1, 2]. Informal caregivers often experience physical and psychological burden, stress, and discomfort [1, 3–7]. Moreover, informal caregiving leads to a restriction of meaningful activities for oneself which affects one’s occupational balance [5, 8, 9].

Occupational balance is defined as a subjective balance between meaningful activities in different life areas, such as self-care, leisure time or productivity. Meaningful activities are characterized by having a specific purpose to a person and include activities a person does, wants to or has to do [10].Occupational balance is of high importance due to its association with health and well-being [11–14]. Its direct and indirect effects on health and quality of life could recently be confirmed [14]. Previous studies identified restricted occupational balance in informal caregivers [5, 8, 9, 15–20] and the need for interventions to improve their occupational balance [5, 8, 9]. Additionally, maintaining or improving informal caregivers’ occupational balance might have positive effects on their health and well-being [9, 20–22]. For example, a study reported an association between parents’ occupational balance and health and well-being of the child they cared for [22].

Therefore, it is important to address and assess occupational balance in informal caregivers. Due to subjectivity of occupational balance, a self-evaluation of one’s occupational balance is needed [23, 24]. Self-reported outcome measures, such as caregiver-reported questionnaires are required for self-evaluation [25]. These outcome measures consider the perspectives of the persons concerned and thus generate outcomes that are meaningful to them [25–28]. Additionally, self-reported outcome measures can be completed regardless of location and without the assistance of health professionals and are therefore inexpensive [29].

Reliable and valid outcome measures are prerequisites to assess deviations of occupational balance of informal caregivers, to set occupational balance interventions and to measure the effectiveness of these interventions [25]. However, self-reported outcome measures must comply with defined measurement properties, such as construct validity, internal consistency, and interpretability, to generate reliable and valid measurement outcomes [25, 30, 31]. Construct validity ensures accordance among scores of the outcome measure and existing knowledge or hypothesis, internal consistency ensures interrelatedness among a scale’s items and interpretability ensures assignment of qualitative meaning in clinical practice [25, 30].

Traditionally, examination of measurement properties has been guided by classical test theory (CTT). However, CTT methods to examine measurement properties have limitations. Item response theory approaches, such as analyses with a Rasch model, have been found to show advantages over CCT [32–35]. The Rasch model defines the probability that a person will answer an item correctly, given a specified person ability and item difficulty. Thus, the Rasch model provides a powerful approach to determine the coherence between the construct to be measured, and the outcome measure [32–34, 36].

Measurement instruments on occupational balance exist. However, these measurement instruments were not specifically developed with and validated in a sample population of informal caregivers [37, 38]. The self-reported questionnaire on Occupational Balance in Informal Caregivers (OBI-Care [37]) is a generic measurement instrument to assess occupational balance in informal caregivers [37]. It was specifically developed with parents of preterm infants, who are considered to be informal caregivers. A German version of the OBI-Care was developed first and subsequently translated into English, only the German version is validated. Previous analyses of the measurement properties of the German version in a sample of parents of preterm infants demonstrated construct validity and internal consistency [37]. However, measurement properties of the German version of the OBI-Care have not been examined in a mixed population of informal caregivers, such as caregivers of persons of different ages and diagnoses [37]. The exploration of its measurement properties in a mixed population of informal caregivers is required to ensure its generic applicability to assess occupational balance in a wider range of informal caregivers.

Thus, the aim of this study was to examine construct validity, internal consistency, and interpretability of the German version of the OBI-Care in a mixed population of informal caregivers.

## Methods

### Design

We conducted a psychometric study, applying a multicenter cross-sectional study design. Measurement properties of the German version of the OBI-Care were analyzed. Specifically, construct validity, internal consistency and interpretability were addressed. This study was part of a larger study, the Occupational Balance Project of Informal caregivers (TOPIC).

### Data collection

From September 2016 to July 2020, numerous strategies were applied to recruit informal caregivers for this multicenter study in Austria. These were personal recruitment in participating centers and self-help groups as well as electronic recruitment through posts on social media (Table 1).

**Table 1:** Recruitment process.

Recruitment type	Participating centers and self-help groups
Personal recruitment (paper survey)	University Hospital Krems, University Hospital St. Pölten, University Hospital Tulln, Hospital Amstetten, Hospital Mistelbach, Hospital Wiener Neustadt, Hospital Zwettl, Rehabilitationcenter Kids Chance Bad Radkersburg, Niederösterreichisches Hilfswerk, self-help groups for informal caregivers of Dachverband für Selbsthilfegruppen Österreich
Online recruitment (electronic survey)	Self-help groups for informal caregivers of Dachverband für Selbsthilfegruppen Österreich

Informal caregivers of persons treated in one of the participating centers and informal caregivers of participating self-help groups were informed about study procedures verbally and in writing by the principal investigator, study assistants, health professionals, including therapists and nurses and self-help group leaders. Subsequently, potential participants were asked to participate in this study and to fill in the paper survey (personal recruitment).

Additionally, informal caregivers were invited electronically to participate in this study. Therefore, the principal investigator, study assistants and self-help group leaders shared written information and a video about study procedures as well as the electronic survey on social media and on the homepages of their institutions (electronic recruitment).

Inclusion criteria were informal caregivers i) who provided informal care for family members, relatives, or friends at the time of participation and ii) with sufficient German reading and writing skills. Exclusion criteria were underaged (≤ 18 years old) informal caregivers. No action was taken to recruit a sample that is representative of the population of informal caregivers in Austria.

Sample size was defined according to recommendations for Rasch analyses, were ten observations (cases) for each item in each category are required, whereby observations do not have to be individual cases [39].

#### Data collection instruments

Participants filled in the paper (personal recruitment) or the electronic (electronic recruitment) survey, digitalized with the program Enterprise Feedback Suite Survey [40], of a set of self-reported questionnaires [41–46] including the German version of the OBI-Care and the following sociodemographic data relevant for this study: informal caregivers’ sex, age, caring effort, caring activities and the number of persons to be cared for as well as sex and age of the persons to be cared for. The OBI-Care consists of 22 items. Each item has a five-choice response scale, ranging from 1, very satisfied to 5, very dissatisfied. Items are summarized in three subscales. Subscale 1 (occupational areas) asks for the satisfaction with the extent of one’s activities. Subscale 2 (occupational characteristics) asks for the characteristics and effects of one’s activities. Subscale 3 (occupational resilience) asks for the adaptability of one’s activities (Table 2). The subscales represent multidimensionality and recently identified dimensions of occupational balance. Sumscores are calculated for each subscale by summating according raw item values [37].

**Table 2:** Subscales and items of the OBI-Care [37].

**Subscale 1**	**Satisfaction with …**
Item_1a	household
Item_1b	caring for others
Item_1c	life management
Item_1d	physical activity / sports
Item_1e	social contacts
Item_1f	health and well-being
Item_1g	leisure
Item_1h	sleep
Item_1i	job, further education and training
**Subscale 2**	**Satisfaction with …**
Item_2a	occupations you do on your own initiative and those you do because of others
Item_2b	usual and unusual daily routines
Item_2c	predictable and unpredictable occupations
Item_2d	important and less important occupations
Item_2e	physically demanding and less physically demanding occupations
Item_2f	mentally demanding and less mentally demanding occupations
Item_2g	indoor and outdoor occupations
**Subscale 3**	**Satisfaction with …**
Item_3a	options to change the order of your occupations
Item_3b	options to spend more time on some occupations and less time on others
Item_3c	options to gather required information to perform new occupations
Item_3d	options to develop required skills to perform new occupations
Item_3e	options to continue to pursue occupations that are meaningful to you
Item_3f	options to find new occupations that are meaningful to you

**Abbreviations:** OBI-Care = Occupational Balance in Informal Caregivers Questionnaire

### Data analyses

Data was entered in a data file and analyzed with the Statistical Package for the Social Sciences (SPSS [47]) and Rasch Unidimensional Measurement Model 2030 (RUMM 2030 [48]). SPSS was used for factor and correlation analyses, RUMM 2030 for analyses with a Rasch Model. Participants who did not fill in the OBI-Care completely were excluded from analyses. Analyses were conducted for each subscale of the OBI-Care. Alpha’s (α) level of significance was set at 0.05. For multiple testing, Bonferroni adjustment was applied [49, 50].

#### Descriptive analyses

Descriptive analyses were carried out to describe sociodemographic data of informal caregivers and persons to be cared. Descriptive analyses included the calculation of means and standard deviations for normal distributed data and medians and interquartile ranges for non-distributed data as well as frequencies and percentages.

#### Examination of psychometric properties

Dimensionality testing and different analyses with a Rasch model were conducted to assess construct validity [34, 51–57]. Dimensionality was examined by factor analyses. Therefore, principal component analysis was applied to extract components and their eigenvalues. Components with eigenvalues ≥ 1 were interpreted as an independent factor. One identified factor was interpreted as unidimensionality of a scale, factors ≥ 2 as multidimensionality. Subscales should be unidimensional to guarantee that the included items measure the same construct [25, 52]. Furthermore, item fit residual statistics and item-trait interaction chi-square statistics were analyzed to determine item fit and overall fit to the Rasch model. Non-significant item fit residuals (-2.5 to 2.5) and a mean item fit residual close to zero with a standard deviation close to one demonstrate an item fit. Non-significant chi-square values with a total chi-square probability value greater than 0.05 indicate overall fit [34, 49, 51, 56, 58, 59]. Moreover, threshold ordering, and the representation of response categories were examined by exploring threshold maps and threshold probability curves. Ordered thresholds indicate that the item’s response categories operate appropriately [34, 49, 51, 56].

Correlation analyses were conducted to assess internal consistency. These were inter-item correlations, item-total correlations, Cronbach’s α and the person separation index (PSI [25, 50]). Inter-item correlations between 0.2 and 0.5 and Cronbach’s α between 0.70 and 0.90 display that items measure the same construct and their appropriate allocation to the scale. Inter-item correlations > 0.7 indicate that the items measure almost the same and one of them might be deleted. Item-total correlations of ≥ 0.3 and a PSI ≥ 0.7 imply that the items discriminate between persons with different abilities [25, 50].

Interpretability was examined by the inspection of floor and ceiling effects [25]. Floor and ceiling effects are displayed when a high proportion (determined as 15%) of the sample population achieves the lowest (nine points for subscale 1, seven points for subscale 2 and six points for subscale 3) or highest score (45 points for subscale 1, 35 points for subscale 2 and 30 points for subscale 3) of an outcome measure. Floor and ceiling effects pose a problem in clinical practice, since persons that already achieved the lowest or highest score at baseline, cannot show any deterioration or improvement at follow up [25, 60].

### Ethical considerations

The current study was approved by the ethics committee of Lower Austria. Participants confirmed their voluntarily participation by returning the paper survey or completing the electronic survey.

## Results

### Participants

In total, 217 informal caregivers participated in this study. Twenty-one participants were excluded due to missing data. Finally, data of 196 informal caregivers were included for analyses, extracted from 107 (55%) electronic surveys and 89 (45%) paper surveys. Sociodemographic data of informal caregivers and persons to be cared for are presented in Table 3. Persons to be cared for had different health conditions and diagnoses, such as cerebral palsy, dementia, cancer, or diabetes.

**Table 3:** Sociodemographic data.

**Informal caregivers**	**Female**	**Male**	**Total**
Sex	171 (87.2%)	25 (12.8%)	196 (100%)
Mean age in years (±SD)	51.5 (±12.0)	57.7 (±15.3)	52.3 (±12.6)
Caring activities for more than one person n (%)	80 (46.8%)	12 (48.0%)	92 (46.9)
Caring effort n (%) ^a^			
low	35 (20.5%)	7 (28.0%)	42 (21.4%)
high	135 (78.9%)	18 (72.0%)	153 (78.1%)
not specified	1 (0.6%)	-	1 (0.5%)
Caring activities n (%) ^b^			
body care and hygiene	138 (80.7%)	17 (68.0%)	155 (79.1%)
household activities	153 (89.5%)	24 (96.0%)	177 (90.3%)
cooking	139 (81.3%)	15 (60.0%)	154 (78.6%)
feeding activities	117 (68.4%)	13 (52.0%)	130 (66.3%)
participation in society, contact with relatives and friends	126 (73.7%)	15 (60.0%)	141 (71.9%)
further activities	83 (48.5%)	15 (60.0%)	98 (50.0%)
**Persons to be cared for**	**Female**	**Male**	**Total**
Sex	104 (52.3%)	90 (47.7%)	194 (99.0%)
Median age in years (IQR)	77.0 (76)	62.0 (61)	68.0 (68)

Abbreviations

^a^ = single answer

^b^ = multiple answers; n = frequency; SD = Standard deviation

### Construct validity

Overall, all subscales of the OBI-Care demonstrated good construct validity. Factor analyses showed that subscale 1 consists of two factors with eigenvalues ≥ 1. Thus, subscale 1 did not satisfy unidimensionality. Subscale 2 and subscale 3 consisted of one component with an eigenvalue ≥ 1 each and therefore complied with unidimensionality (Table 4).

**Table 4:** Dimensionality.

Subscale 1						Subscale 2					Subscale 3				
Item	Eigenvalue^a^			C^a^		Item	Eigenvalue			C	Item	Eigenvalue			C
	**total**	**% of VA**	**CUM %**	**1**	**2**		**total**	**% of VA**	**CUM %**	**1**		**total**	**% of VA**	**CUM %**	**1**
Item_1a	4.438	49.313	49.313	0.610	0.636	Item_2a	3.976	56.796	56.796	0.769	Item_3a	3.995	66.582	66.582	0.779
Item_1b	1.164	12.933	62.246	0.590	0.626	Item_2b	0.796	11.366	68.162	0.777	Item_3b	0.710	11.836	78.418	0.813
Item_1c	0.799	8.874	71.12	0.681	0.263	Item_2c	0.589	8.409	76.571	0.694	Item_3c	0.532	8.875	87.293	0.812
Item_1d	0.610	6.776	77.896	0.709	-0.276	Item_2d	0.497	7.093	83.664	0.788	Item_3d	0.278	4.628	91.921	0.809
Item_1e	0.477	5.301	83.197	0.783	-0.26	Item_2e	0.447	6.388	90.052	0.756	Item_3e	0.264	4.400	96.321	0.841
Item_1f	0.455	5.060	88.258	0.771	-0.229	Item_2f	0.370	5.279	95.330	0.717	Item_3f	0.221	3.679	100	0.840
Item_1g	0.375	4.172	92.430	0.743	-0.082	Item_2g	0.327	4.670	100	0.769					
Item_1h	0.368	4.085	96.515	0.707	-0.163										
Item_1i	0.314	3.485	100	0.701	-0.263										

Abbreviations

^a^ = extraction method: principal component analysis; C = components; CUM = cumulative; VA = Variance

For all subscales, item fit residuals ranged between -2.5 and +2.5 and mean item fit residuals were close to zero with a standard deviation close to one. Chi square probability values for each subscale were greater than 0.05. Therefore, all values indicated item fit and overall fit to the Rasch model. Detailed results of Rasch analyses are provided in Table 5.

**Table 5:** Rasch analyses.

**Subscale 1**	**mean item fit** 0.267 (± 0.997)			**chi-square probability** 0.383	
	**item statistics** ^**a**^			**fit statistics** ^**a**^	
Items	location	SE	residual*	chi-square ^b^**	f-statistics ^b^
Item_1a	0.682	0.097	0.861	0.965	0.457
Item_1b	0.704	0.091	1.993	3.432	1.584
Item_1c	0.441	0.082	0.263	1.377	0.541
Item_1d	-0.345	0.083	0.194	1.569	0.773
Item_1e	-0.163	0.081	-1.188	4.036	3.002
Item_1f	-0.687	0.082	-1.062	4.586	3.286
Item_1g	-0.445	0.083	-0.173	2.328	1.240
Item_1h	-0.048	0.076	0.638	0.146	0.080
Item_1i	-0.140	0.079	0.904	0.702	0.287
**Subscale 2**	**mean item fit** 0.406 (± 0.792)			**chi-square probability** 0.517	
	**item statistics** ^**a**^			**fit statistics** ^**a**^	
Items	location	SE	residual*	chi-square ^c^**	f-statistics ^c^
Item_2a	-0.361	0.098	0.483	2.592	1.406
Item_2b	-0.049	0.106	-0.56	3.584	2.332
Item_2c	-0.245	0.102	1.315	1.223	0.603
Item_2d	-0.419	0.105	-0.028	1.653	1.060
Item_2e	0.200	0.098	0.184	0.855	0.452
Item_2f	0.495	0.097	1.608	2.265	1.098
Item_2g	0.379	0.099	-0.161	0.946	0.537
**Subscale 3**	**mean item fit** 0.076 (± 0.615)			**chi-square probability** 0.707	
	**item statistics** ^**a**^			**fit statistics** ^**a**^	
Items	location	SE	residual*	chi-square ^d^**	f-statistics ^d^
Item_3a	0.054	0.104	1.068	1.656	0.710
Item_3b	-0.191	0.111	0.166	0.242	0.173
Item_3c	0.401	0.103	0.242	1.676	0.797
Item_3d	0.212	0.102	0.139	0.248	0.145
Item_3e	-0.010	0.102	-0.491	1.602	1.027
Item_3f	-0.466	0.097	-0.664	3.517	2.422

Abbreviations

^a^ = rounded to three decimals

^b^ = Bonferroni adjusted probability level = 0.001111

^c^ = Bonferroni adjusted probability level = = 0.007143

^d^ = Bonferroni adjusted probability level = 0.001667

* = Deviations from the recommended range of -2.5 to +2.5 indicating item misfit are bold

** = Bonferroni adjusted statistically significant deviations indicating overall misfit are bold; p = probability; SE = Standard error

All items of each subscale showed ordered thresholds. Additionally, all response categories were represented (Fig 1).

**Fig 1:** Ordered thresholds indicate that the item’s response categories operate appropriate.

### Internal consistency

Except for three item pairs of subscale 3, all items satisfied criteria for inter-item correlations (< 0.70). Inter-item correlations for item 3a and item 3b, item 3c and item 3d as well as for item 3e and item 3f indicated redundancy among the items (> 0.70). However, these items were only statically redundant but not related to their content. Additionally, all items showed good item-total correlations (> 0.3), Cronbach’s α (0.7 to 0.9) and person separation indices (> 0.7). Thus, all subscales demonstrated internal consistency. Detailed results are presented in Table 6.

**Table 6:** Correlation analyses, PSI and Cronbach’s α.

**Sub-scale 1**	**Inter-Item Correlation** ^*^									**PSI**	**Cronbach‘s α**
										0.861	0.868
Item	Item_1a	Item_1b	Item_1c	Item_1d	Item_1e	Item_1f	Item_1g	Item_1h	Item_1i	**Total-Item Correlation**	**Cronbach’s α if item deleted**
Item_1a	1.000	0.559	0.486	0.306	0.309	0.305	0.368	0.356	0.291	0.515	0.861
Item_1b	0.559	1.000	0.430	0.232	0.338	0.307	0.314	0.302	0.262	0.467	0.865
Item_1c	0.486	0.430	1.000	0.450	0.482	0.415	0.354	0.325	0.419	0.589	0.855
Item_1d	0.306	0.232	0.450	1.000	0.615	0.551	0.452	0.400	0.388	0.613	0.852
Item_1e	0.309	0.338	0.482	0.615	1.000	0.597	0.468	0.457	0.539	0.695	0.844
Item_1f	0.305	0.307	0.415	0.551	0.597	1.000	0.580	0.485	0.483	0.680	0.846
Item_1g	0.368	0.314	0.354	0.452	0.468	0.580	1.000	0.535	0.435	0.633	0.850
Item_1h	0.356	0.302	0.325	0.400	0.457	0.485	0.535	1.000	0.519	0.606	0.854
Item_1i	0.291	0.262	0.419	0.388	0.539	0.483	0.435	0.519	1.000	0.603	0.853

**Sub-scale 2**	**Inter-Item Correlation** ^*^							**PSI**	**Cronbach‘s α**
								0.871	0.870
Item	Item_2a	Item_2b	Item_2c	Item_2d	Item_2e	Item_2f	Item_2g	**Total-Item Correlation**	**Cronbach’s α if item deleted**
Item_2a	1.000	0.632	0.442	0.550	0.428	0.460	0.504	0.662	0.850
Item_2b	0.632	1.000	0.574	0.554	0.442	0.406	0.469	0.679	0.848
Item_2c	0.442	0.574	1.000	0.485	0.445	0.383	0.400	0.590	0.859
Item_2d	0.550	0.554	0.485	1.000	0.501	0.453	0.520	0.676	0.848
Item_2e	0.428	0.442	0.445	0.501	1.000	0.539	0.600	0.651	0.851
Item_2f	0.460	0.406	0.383	0.453	0.539	1.000	0.526	0.605	0.858
Item_2g	0.504	0.469	0.400	0.520	0.600	0.526	1.000	0.668	0.849

**Sub-scale 3**	**Inter-Item Correlation** ^*^						**PSI**	**Cronbach‘s α**
							0.858	0.897
Item	Item_3a	Item_3b	Item_3c	Item_3d	Item_3e	Item_3f	**Total-Item Correlation**	**Cronbach’s α if item deleted**
Item_3a	1.000	**0.739**	0.548	0.483	0.519	0.555	0.680	0.886
Item_3b	**0.739**	1.000	0.545	0.478	0.594	0.622	0.723	0.881
Item_3c	0.548	0.545	1.000	**0.728**	0.566	0.573	0.719	0.881
Item_3d	0.483	0.478	**0.728**	1.000	0.639	0.599	0.712	0.882
Item_3e	0.519	0.594	0.566	0.639	1.000	**0.747**	0.754	0.875
Item_3f	0.555	0.622	0.573	0.599	**0.747**	1.000	0.759	0.875

Abbreviations

* = inter-item correlations > 0.7 showing redundancy are bold; α = Alpha; PSI = person separation index

### Interpretability

Exploration of floor and ceiling effects indicated interpretability. No significant floor and ceiling effects were found. For subscale 1, one (0.6%) person of the sample population achieved the lowest score (9) and the highest score (45). For subscale 2, none (0.0%) of the participants reached the lowest score (7) and two (1.1%) reached the highest score (35). For subscale 3, two (1.1%) persons scored the lowest score (6) and three (1.7%) the highest score (30).

## Discussion

Within this study we examined psychometric properties of the German version of the OBI-Care in a sample population of informal caregivers.

Construct validity and internal consistency of the German version of the OBI-Care have already been examined in one of our previous studies [37]. However, the results of both studies differ partly and to our knowledge this is the first time that measurement properties of the OBI-Care have been examined in another population of informal caregivers.

As part of construct validity, we identified multidimensionality of subscale 1. This result does not comply with results of our previous studies, where subscale 1 displayed to be unidimensional [37]. However, it should be pointed out that we interpreted components with eigenvalues ≥ 1 as an independent factor. There is no uniform definition as to which value the eigenvalue has to exceed to be defined as a factor [25]. In other studies eigenvalues are defined as an independent factor from ≥ 3 onwards [55, 61]. Taking this definition into account, subscale 1 would consist of only one factor and be unidimensional. Additionally, to our knowledge the OBI-Care is the first occupational balance measure that considers multidimensionality of occupational balance in terms of measurement properties by using subscales [24, 37]. Thus, further analyses on the subscales of the OBI-Care are warranted.

Examination of internal consistency indicated that item 3a on changed chronology and item 3b on adapted time expenditure as well as item 3e on perpetuating occupations and item 3f on finding new occupations were statistically redundant. This result differs from our previous study [37]. It is possible that it is not important for informal caregivers which kind of meaningful occupations and in which order or amount of time they are performed, as long as the performance is possible. Inter-item correlations for item 3c on knowledge gathering and item 3d on skills acquisition indicated redundancy as well. Within our previous study we came to the same conclusion [37]. Thus, we believe that participants do not differ between knowledge gathering and skills acquisition. Supplementing these items with an example might enhance comprehensibility of the items.

Since occupational balance is a latent construct, it cannot be assessed directly [23]. Additionally, there is no consent how to assess occupational balance. In line with other existing occupational balance measures [62, 63], items of the OBI-Care ask for satisfaction with manifest components of occupational balance. Another occupational balance measure asks for the ability to perform manifest components of occupational balance [23]. Lack of consensus on the conceptualization and dimensions of occupational balance [24, 64] leads to inconsistent occupational balance measures and uncertainty how to measure occupational balance. Therefore, further studies on the conceptualization and dimensions of occupational balance are required.

The examination of interpretability of the OBI-Care is novel and thus provides new findings on the application of the OBI-Care in clinical practice. However, by calculating floor and ceiling values we determined the OBI-Care’s capability to measure the full range of occupational balance exclusively. Further explorations on interpretability, such as cut off values and minimal important change are recommended [25, 37].

Previous studies indicate that caregivers’ occupational balance and the engagement in meaningful activities might have an impact on caregivers’ subjective health and wellbeing as well as on subjective health and well-being of the persons to be cared for [5, 8, 9, 20, 21]. Thus, it is recommended that health professionals, such as occupational therapists, support informal caregivers’ engagement in meaningful activities and thereby strengthen their occupational balance.

### Strengths and limitations

This study shows several strengths and limitations. Construct validity, internal consistency, and interpretability present essential components of psychometric properties. However, further studies are warranted to examine other psychometric properties, such as responsiveness [25]. The examination of psychometric properties using analyses with a Rasch model facilitates the identification of measurement inadequacies that might not be detected by classical test theory and thus provides a powerful alternative [32–34].

We examined psychometric properties in a mixed sample population of informal caregivers to ensure applicability independent of the caregivers. The examination of measurement properties might be replicated in diverse populations characterized by informal caregivers of people with specific diagnoses, such as dementia. We examined psychometric properties of the German version of the OBI-Care exclusively. Therefore, an examination of the existing English version of the OBI-Care [37] is required.

Additionally, the multicenter design and numerous recruitment strategies led to a high diversity of persons to be cared for. However, it should be noted that 87.2% of informal caregivers included in this study were female. Analyses within a sample with more male informal caregivers might differ. Differences in the burden perceived by female and male informal caregivers have been identified previously [65]. Additionally, occupational balance has been found to differ in women and men [66, 67]. Moreover, our study supports findings of previous studies that informal care is still mainly provided by women [68, 69] and thus indicate the consideration of gender specific research on informal caregivers. Furthermore, it has to be considered that the application of numerous recruitment strategies (personal and online recruitment) may have led to potential bias [70].

## Conclusion

The German version of the OBI-Care demonstrates construct validity, internal consistency, and interpretability. Thus, the OBI-Care can be applied to measure occupational balance in informal caregivers and to assess effectiveness of occupational balance interventions for informal caregivers.
